# Waterloo Handedness Questionnaire: Cross-Cultural Adaptation and Psychometric Properties of the Arabic Version

**DOI:** 10.1155/2022/3026415

**Published:** 2022-10-12

**Authors:** Saleh M. Aloraini

**Affiliations:** Department of Physical Therapy, College of Medical Rehabilitation, Qassim University, Saudi Arabia

## Abstract

Handedness is one of the most studied behavioural predictors of cerebral lateralization. Assessing handedness is often essential in neuropsychology and motor behaviour research. Thus, it is important that self-reported assessment tools for determining handedness are available in multiple languages for different cultures. The purpose of the present study was to conduct a translation and cross-cultural adaptation of the Waterloo Handedness Questionnaire into the Arabic language and to assess its psychometric properties. Two independent forward translations were performed by two native Arabic speakers and then synthesized into one version. The synthesized version was backtranslated into English by two independent bilingual translators. An expert committee was formed to review the translation and adaptation process. A final Arabic version of the WHQ was obtained, the WHQ-Ar. Two hundred and ninety adult Arabic speakers were recruited to participate in the study and investigate the properties of the WHQ-Ar. Results showed that the WHQ-Ar had no floor or ceiling effect. For construct validity, results of factor analysis revealed that the WHQ-Ar had two dimensions. Further, the WHQ-Ar had excellent internal consistency with Cronbach′s alpha = 0.93. For test-retest reliability, intraclass correlation coefficient score was 0.94. The Bland-Altman plot showed acceptable agreement between test and retest scores. Therefore, the WHQ-Ar is a valid, reliable tool and ready for use among the Arabic-speaking population for determining handedness.

## 1. Introduction

Cerebral lateralization refers to the preferred use of one side of the body with regard to hands, feet, eyes, and ears [1]. Hand preference, or handedness, is one of the most studied behavioural predictors of cerebral lateralization [1]. Assessing handedness is often essential in neuropsychology and motor behaviour research. Historically, information on handedness has been obtained via observation, self-reporting, or by using survey questionnaires [2]. Of the three methods, survey questionnaires are considered to be the most reliable as all respondents answer the same questions [2]. Further, survey questionnaires account for the degree of handedness rather than dichotomizing handedness into either left-handed or right-handed. As suggested in previous research, asking singular questions to categorize handedness does not correlate well with actual hand preference [3–5].

Research related to handedness has given rise to the multiple theories that attempt to explain limb dominance, among them is the dynamic dominance hypothesis [6]. The dynamic dominance hypothesis of motor lateralization suggests that among individuals with right hand preference, the left cerebral hemisphere specializes in predictive processes that are aimed at achieving smooth and efficient movement under mechanically stable conditions. On the other hand, the right hemisphere specializes in impedance control that aim for robustness of movement performed under unpredictable and mechanically unstable conditions [6, 7]. As such, the dynamic dominance hypothesis stipulates that the advantage seen in the preferred hand is in the anticipation and utilization of the dynamics of movement across multiple segments. Conversely, the less preferred hand has the advantage of controlling postural errors, most notably the final limb state (e.g., goal-directed movements).

Assessing handedness is important as hand preference often correlates with other lateralized functions, such as cerebral lateralization of language and lateralization of visuospatial abilities [8]. Further, assessing handedness provides valuable information for clinicians working in the field of rehabilitation. For example, following stroke rehabilitation interventions primarily emphasize stimulation of the recovery of the sensorimotor function of the paretic upper extremity. The other upper extremity, commonly termed the unaffected upper extremity, is often considered a reference point. Therefore, it is assumed that this side has no deficit. However, previous research has shown that the “unaffected” upper extremity may suffer from subtle deficits [9–15]. The changes seen in the “less-affected” upper extremity can be the results of damage to either the dominant or nondominant cerebral hemisphere.

Previous research reports that damage to the dominant hemisphere (i.e., hemisphere contralateral to the dominant hand) results in impairments to initial ballistic component of reaching movement, but not to the secondary slower component [16]. However, individuals with damage to the nondominant hemisphere did not show impairment in this aspect of movement but showed greater deficits in tasks with high-precision requirements [16]. Moreover, previous research has reported that people after stroke respond differently to rehabilitation therapy according to which cerebral hemisphere has the lesion (dominant vs. nondominant), which was assessed using hand preference. Results showed that there was a clear advantage following therapy for individuals with lesions in the dominant hemisphere [17, 18]. Assessing handedness among individuals poststroke aids in understanding the different impairments among individuals with dominant hemisphere lesions and those with nondominant hemisphere lesions, thus providing rehabilitation care efficiently and more effectively based on the side of stroke.

There are a plethora of instruments used to assess handedness, among them is the Waterloo Handedness Questionnaire (WHQ) [19]. The WHQ is a multi-item (36 questions), self-reported handedness questionnaire. This questionnaire is one of the most used instruments to assess handedness and is easy to use and interpret [20]. The questions in the WHQ are answered on a 5-level, Likert-type scale to determine the degree of preferred hand use. Responses to each question are assigned a value between -2 and 2, with scores closer to 0 reflecting equal hand preference, scores closer to -2 indicating left hand preference, and 2 indicating right hand preference. The sum of the total WHQ scores can be used to categorize a respondent as left-handed (score of -24 or less), mixed-handed (score of -23 to +23), or right-handed (score of +24 or higher).

As mentioned above, assessing handedness is of great importance in neuropsychology and motor behaviour research. Further, determining handedness is valuable for clinicians working in the field of rehabilitation and motor training. The WHQ has not been translated and cross-culturally adapted to the Saudi population. Thus, the purpose of the current study is to translate the WHQ to the Arabic language, adapt it to our culture, and investigate its validity and reliability.

## 2. Methods

### 2.1. Study Design

This is a longitudinal study that is aimed at cross-culturally adapting the WHQ into Arabic. The guidelines for the cross-cultural adaptation of self-reported measures by Beaton and colleagues were followed [21]. Prior to the commencement of our study, Dr. Lorin Elias, who is one of the researchers who developed the WHQ, was contacted to obtain permission to translate the questionnaire. The local Research Ethics Committee approved all procedures. All participants provided an informed consent.

### 2.2. Participants and Recruitment

Recruitment was carried out in the community via advertisement posters and word of mouth. Participants were included if they were adults (≥18 years of age) with typical motor performance and able to read, speak, and understand Arabic. Participants were excluded if they were unable to read or speak Arabic. Recruitment of participants was carried out in all regions of Saudi Arabia. Sample size for the study was based on recommendations for factor analyses, which range from 3 to 10 subjects per variable (item) of the questionnaire, with a minimum of 50 participants in total [22]. The current study is aimed at recruiting eight subjects per the WHQ 36 items.

### 2.3. Procedures

The process started with translating the WHQ into Arabic. Two native Arabic speakers independently forward translated the WHQ into Arabic. Afterwards, the two translations were synthesized into one version. The synthesized version was then backtranslated into English by two independent bilingual translators. Subsequently, an expert committee was formed and consisted of two methodologists and two language professionals and all forward and backward translators to review the translation and adaptation process of the WHQ. The expert committee suggested minor linguistic and idiomatic changes and reached a consensus that the reproduced backtranslated English version of the culturally adapted WHQ was compatible with the original one. Thus, the prefinal version of the Arabic translated WHQ was created and ready to be field-tested with participants.

A pilot study was conducted to examine the prefinal version of the Arabic WHQ on a sample of 30 participants who match the recruitment criteria. Participants in the pilot testing were asked to independently complete the questionnaire and respond freely and honestly to all items. Participants were then briefly interviewed independently to ask them on how well they understood the completed questionnaire. Following the 30-participant pilot testing, the final Arabic version of the Waterloo Handedness Questionnaire (WHQ-Ar) was produced.

The WHQ was then field-tested to further evaluate its psychometric properties, including validity, reliability, and internal consistency. Participants who matched the recruitment criteria provided a written informed consent. Subsequently, participants were asked to complete a general information sheet for demographic data. The information sheet also included a commonly used question to assess handedness “which hand do you use to write with a pen?,” with two options “right” or “left.” Lastly, in order to assess test-retest reliability, participants were asked to complete the WHQ-Ar twice, with a period of one-week apart. The period of one week for assessing test-retest reliability was determined based on previous recommendations [23].

### 2.4. Data Analyses

Data analysis included descriptive statistics for participants' characteristics and hand dominancy as assessed by the handwriting question and by the WHQ-Ar. Face validity was determined during the piloting process via participants' responses to the interview questioning the relevance and appropriateness of the WHQ-Ar to determine hand dominancy. Content validity was established by the consensus of the expert committee members regarding the relevance and appropriateness of the WHQ-Ar to determine the handedness for Arabic speakers. Floor and ceiling effects of the WHQ-Ar were determined by computing the percentage of participants scoring the lowest or highest on the WHQ-Ar. The WHQ-Ar was considered to have a floor or ceiling effect when more than or equal to 15% of the participants had the lowest or highest possible score.

Construct validity of the WHQ-Ar was determined using factor analysis with direct oblimin rotation method to extract factors of eigenvalues greater than Kaiser's criterion of one [24]. To assess the internal consistency of the WHQ-Ar, Cronbach's *α* was used with a score of 0.7 considered as the minimum score for an adequate consistency. Intraclass correlation coefficient for absolute agreement (ICC 2,1) was used to assess test-retest reliability, and a minimum value of 0.7 was set for an adequate test-retest reliability of the WHQ-Ar. Standard error of measurement (SEM) was used to examine the WHQ-Ar measurement error associated with test-retest.

To assess construct validity, hypothesis testing was used. The WHQ-Ar was hypothesized to have moderate to strong positive correlation (rho ≥ 0.4) with the hand-dominancy question answered by participants (handwriting). Spearman's rho was used to determine the hypothesized correlation for construct validity. All analyses were performed using IBM SPSS statistical software, version 26 (IBM Corp. Armonk, NY). Significance was set at *α* = 0.05.

## 3. Results

Two hundred and ninety Arabic speakers participated in this study.  Table 1 shows the characteristics of participants. The overall process of the translation and cross-cultural adaptation of the WHQ-Ar was straight forward with no issues. One of the changes recommended by the expert committee following the pilot was to change the answering grid (La, Lu, Eq, Ra, and Ru) of the WHQ and not use abbreviations for the Arabic language and use full description (left always, left usually, equal use, right always, and right usually) for better clarity of the WHQ-Ar. Additionally, individuals who were interviewed following the pilot study stated that the questionnaire was clear, relevant, and appropriate to determine hand dominancy. The testament of these individuals supports the face validity of the WHQ-Ar. Regarding content validity, the expert committee reached consensus regarding the relevance and appropriateness of the WHQ-Ar for Arabic speakers for determining hand dominancy. Moreover, the completeness of the WHQ-Ar items was satisfactory and the absence of floor and ceiling effects in the analysis further supports the WHQ-Ar content validity.

For construct validity, the Kaiser-Meyer-Olkin measure of sampling adequacy was met (*p* = 0.98) and Bartlett's test of sphericity was satisfied (*χ*_45_^2^ = 10469.13, *p* < 0.001). These findings support the appropriateness for utilizing factor analysis. Exploratory factor analysis indicated that two factors had an eigenvalue greater than Kaiser's criterion of one, factor 1 = 21.58 and factor 2 = 2.20. Combined, these two factors explain 66.07% of the variance (Table 2). Following extraction, these two factors explained 64.14% of the variance. Nonetheless, it is reasonable to accept that all items have one dimension. The rationale for considering one dimension for all items can be attributed to two reasons. First, the sum of the second factor's eigenvalue after extraction (1.83) is drastically less than the first factor (21.26) (Figure 1). Second, the loading of items on the second factor were all less than 0.3. However, loading of items for the first factor were all ≥0.5 and ranged from 0.506 to 0.906 (Table 3).

Results of internal consistency analysis showed that the WHQ-Ar has excellent internal consistency with Cronbach's *α* = 0.979. In regard to WHQ-Ar stability, results showed excellent test-retest reliability with an ICC = 0.976 (95%CI = 0.969-0.981). The Bland-Altman plot showed acceptable agreement between test and retest scores (Figure 2). For scale measurement error assessed from test-retest, the SEM = 9.2 points. Lastly, the hypothesized correlation between the WHQ-Ar and the participants' hand dominancy assessed via the handwriting question was significant with rho = 0.47, *p* < 0.001.

## 4. Discussion

The present study is aimed at translating and culturally adapting the WHQ into the Arabic language and reporting on the psychometric properties of the WHQ-Ar. The overall findings of the study indicate that the translation and cultural adaptation of the WHQ into the WHQ-Ar were successful. Further, the measurement properties including validity, internal consistency, test-retest reliability, and measurement error of the WHQ-Ar were excellent and support its use as a measure of handedness.

During the translation and cross-cultural adaptation phase of the study, only one change was made to the questionnaire. The change in the questionnaire involved changing the answering grid to use the full description of answers rather than using abbreviations. This change in the answering grid was recommended and agreed upon by the expert committee involved in the study for the purpose of improving the clarity of the WHQ-Ar for Arabic speakers. One of the reasons for omitting the abbreviations from the questionnaire was related to the Arabic language itself, as using abbreviations is uncommon in Arabic.

The face validity of the WHQ-Ar is supported by the testaments of the participants involved in the study and by the consensus of the expert committee. Both parties reported that the WHQ-Ar is clear, relevant, and appropriate for assessing handedness. Moreover, the consensus of the expert committee mentioned above also supports the content validity of the WHQ-Ar. In addition, the absence of floor and ceiling effects of the WHQ-Ar indicates that it has adequate content validity [23]. For concurrent validity, handedness was assessed using another commonly used tool. Participants were asked “which hand do you use to write with a pen?” This question is commonly used to assess hand preference and was previously reported as a method to assess self-reported handedness [25]. The results of the study show that the WHQ-Ar was significantly related to the handwriting question used in the present study. Thus, the WHQ-Ar can assess handedness similarly to the handwriting question. Results of construct validity show that factor analysis of the WHQ-Ar indicates that all factors had significant loadings with two main factors (skilled and unskilled activities). This finding is similar to previous studies reporting on the cross-cultural adaptation of the WHQ [26].

The internal consistency of the WHQ-Ar was excellent with Cronbach's *α* = 0.93, indicating that items within the questionnaire are correlated, homogenous, and not redundant [27]. Cronbach's *α* of the WHQ-Ar did not change with deletion of items one at a time (Table 3). As such, the consistency of Cronbach's *α* indicates that all items are homogenous and correlated well with each other and that removal of any item would not improve the internal consistency and homogeneity of the scale. Similarly, reliability analysis of the WHQ-Ar showed that it has excellent test-retest reliability with ICC = 0.976. The magnitude of reliability found in the present study is higher than previously reported [26]. In regard to SEM, which was 9.2 points, when expressed as a percentage of the overall WHQ-Ar score, SEM was 6.3%. The SEM, based on its value and percentage relative to the overall score, the measurement error of WHQ-Ar found in this study indicates excellent reliability. Furthermore, the findings of the Bland-Altman plot showed adequate agreement between test and retest scores, with over 95% of the scores between the agreement lines, indicating excellent reliability of the WHQ-Ar.

The translation and cross-cultural adaptation of the WHQ into the Arabic language performed in this study are extremely important to researchers, clinicians, and practitioners who work in the field of motor learning and training within the Arabic-speaking world. There is a need for a tool with sound psychometric properties that can assess handedness. The findings in the current study show that the WHQ-Ar is a valid and reliable tool for assessing handedness. As mentioned above, survey questionnaires account for the degree of handedness rather than dichotomizing handedness into either left- or right-handed. Previous research suggests that handedness falls into a spectrum rather than either left or right [1, 28–37].

Participants recruited in the current study were all from Saudi Arabia. However, the translation of the WHQ was performed into modern standard Arabic language without the use of any local dialects. As such, the WHQ-Ar can be used in all other Arabic-speaking countries as modern standard Arabic language is used and understood in these countries. Furthermore, the participants recruited in the current study are all adult, non-disabled individuals. Further research is encouraged to examine the characteristics of the WHQ-Ar among different populations.

## 5. Conclusion

In conclusion, this study was carried out to culturally adapt the WHQ and to examine measurement properties of the Arabic version of this questionnaire. The adaptation process was smooth with slight modification to the original WHQ. The WHQ-Ar is a valid and reliable measure for determining handedness. These measurement properties of the WHQ-Ar affirm the usefulness of this measure for all practical and research purposes.

## Figures and Tables

**Figure 1:** Exploratory factor analysis figure showing the factor number on the horizontal axis and the eigenvalue on the vertical axis.

**Figure 2:** Bland-Altman plot.

**Table 1:** Participants' characteristics; *n* = 290.

Age in years (mean ± SD)	29.9 ± 11.3
Gender	
Male	133 (45.9%)
Female	157 (54.1%)
Education status	
No education	1 (0.3%)
Elementary	5 (1.7%)
Intermediate	19 (6.6%)
High school	103 (35.5%)
University graduate	150 (51.7%)
Higher education	12 (4.1%)
Employment status	
Student	132 (45.5%)
Employed	101 (34.8%)
Unemployed	57 (19.7%)
Dominant hand^∗^	
Left	26 (9.0%)
Right	264 (91.0%)

^∗^Dominant hand was assessed based on answering the question: “*which hand do you use to write with a pen?*”.

**Table 2:** WHQ-Ar factor structure.

Factor	Initial eigenvalue			After extraction		
	Total	% of variance	Cumulative %	Total	% of variance	Cumulative %
1	21.58	59.95	59.95	21.26	59.06	59.06
2	2.20	6.12	66.07	1.83	5.08	64.14
3	0.95	2.64	68.71			
4	0.85	2.35	71.06			
5	0.78	2.15	73.22			
6	0.70	1.95	75.16			
7	0.58	1.61	76.77			
8	0.57	1.59	78.37			
9	0.54	1.51	79.87			
10	0.53	1.47	81.34			
11	0.50	1.39	82.74			
12	0.49	1.35	84.08			
13	0.43	1.20	85.29			
14	0.42	1.17	86.46			
15	0.39	1.08	87.54			
16	0.38	1.06	88.60			
17	0.35	0.97	89.57			
18	0.34	0.93	90.50			
19	0.32	0.88	91.38			
20	0.31	0.85	92.23			
21	0.29	0.82	93.05			
22	0.28	0.77	93.82			
23	0.25	0.71	94.52			
24	0.23	0.64	95.16			
25	0.21	0.58	95.75			
26	0.20	0.56	96.30			
27	0.19	0.53	96.83			
28	0.18	0.49	97.32			
29	0.17	0.46	97.78			
30	0.15	0.40	98.19			
31	0.14	0.38	98.57			
32	0.13	0.36	98.93			
33	0.12	0.32	99.25			
34	0.11	0.31	99.56			
35	0.07	0.24	99.80			
36	0.07	0.20	100.00			

**Table 3:** Internal consistency, rotated factor loadings for the WHQ-Ar 36 items using principal axis method with the explained variance for the factor, *n* = 290.

Questionnaire (single factor)	Cronbach's *α*	Items	Cronbach's *α* if item deleted	Factor loadings
Handedness	0.979	Item 1	0.979	0.729
		Item 2	0.978	0.867
		Item 3	0.979	0.665
		Item 4	0.979	0.720
		Item 5	0.978	0.868
		Item 6	0.978	0.879
		Item 7	0.979	0.741
		Item 8	0.978	0.883
		Item 9	0.978	0.884
		Item 10	0.979	0.619
		Item 11	0.978	0.857
		Item 12	0.978	0.768
		Item 13	0.978	0.850
		Item 14	0.979	0.761
		Item 15	0.978	0.906
		Item 16	0.978	0.766
		Item 17	0.980	0.635
		Item 18	0.979	0.515
		Item 19	0.979	0.506
		Item 20	0.980	0.548
		Item 21	0.979	0.712
		Item 22	0.979	0.744
		Item 23	0.978	0.863
		Item 24	0.978	0.888
		Item 25	0.979	0.754
		Item 26	0.979	0.723
		Item 27	0.978	0.869
		Item 28	0.979	0.693
		Item 29	0.978	0.868
		Item 30	0.978	0.868
		Item 31	0.979	0.654
		Item 32	0.978	0.806
		Item 33	0.978	0.818
		Item 34	0.979	0.733
		Item 35	0.979	0.679
		Item 36	0.979	0.754

## Data Availability

The data used to support the findings of this study are available from the corresponding author upon request.
